# Recycle the dental fairy’s package: overview of dental pulp stem cells

**DOI:** 10.1186/s13287-018-1094-8

**Published:** 2018-12-13

**Authors:** Xianrui Yang, Li Li, Li Xiao, Donghui Zhang

**Affiliations:** 1 Department of Orthodontics, State Key Laboratory of Oral Disease, National Clinical Research Center for Oral Diseases, West China Hospital of Stomatology, Sichuan University, Chengdu, 610041 China; 2 Department of Stomatology, Sichuan Academy of Medical Science & Sichuan Provincial People’s Hospital, Chengdu, 610072 China; 3 State Key Laboratory of Biocatalysis and Enzyme Engineering, School of Life Science, Hubei University, Wuhan, 430062 Hubei China

## Abstract

Adult stem cells are excellent cell resource for cell therapy and regenerative medicine. Dental pulp stem cells (DPSCs) have been discovered and well known in various application. Here, we reviewed the history of dental pulp stem cell study and the detail experimental method including isolation, culture, cryopreservation, and the differentiation strategy to different cell lineage. Moreover, we discussed the future potential application of the combination of tissue engineering and of DPSC differentiation. This review will help the new learner to quickly get into the DPSC filed.

## Background

Stem cell (SC) was firstly termed and reported in the literature in the nineteenth century by Alexander Maksimov [64]. During the advancement of the stem cell filed, various types of stem cells were discovered in different tissues including dental pulps. One of them called dental pulp stem cells (DPSCs) were discovered by Dr. Irina Kerkis as adult stem cells in 2005, and then immature dental pulp stem cells (IDPSCs) were discovered through dental pulp organ culture as a pluripotent subpopulation of DPSCs in 2006 [34]. Bone marrow stem cells (BMSCs) were derived from the bone marrow, which was the most widely studied stem cell. As not one kind of BMSCs, DPSCs were derived from the dental pulp but not from the bone marrow. Researches have been trying to compare the differences between them. Kim et al. focused on exploring the gene expression profile in DPSCs and BMSCs by Gene expression analysis and found different upregulated and downregulated transcripts in DPSCs compared to BMSCs [35]. Kumar et al. focused on the secretome of neurogenic potential of DPSCs and BMSCs, pointed out that DPSCs was a better stem cell sources in neural lineage differentiation [38]. Moreover, Tamaki et al. compared the proliferative and clonogenic potentials between DPSCs and BMSCs, claiming that the DPSCs from the teeth possessed greater proliferative potential [71]. When comparing the odontogenic capability, DPSCs showed more striking odontogenic capability than BMSCs, which suggested more suitable candidate cells for tooth regeneration [86].

The two shining points of SC are its pluripotency and differentiation ability, so as DPSCs. The DPSCs have high proliferative potential which shows a strong cloning ability, originating from dental pulp genesis (Fig. 1) [83, 89]. During the development, the dental pulp consists of both mesenchymal and ectodermic components, including neural crest cells with plasticity and multipotential ability. Researchers compared DPSCs with stem cells from human exfoliated deciduous (SHEDs) and bone marrow stem cells (BMSCs) finding that DPSCs showed a more mature phenotype than SHEDs [19] and higher proliferation rate than BMSCs [52]. More recent studies indicated that DPSCs may exist in perivascular areas [67].

**Fig. 1:** Dental pulp stem cell origins and applications

The most obvious advantages of DPSCs are its highly proliferative capacity and differentiation possibility into various cells including epithelial cells, vascular cells, adipocytes, odontoblasts, osteoblasts, neuronal cells, and muscular cells. As the dental pulp is one of the major sites when considering bone marrow as the choice for hematopoietic stem cell collection, DPSCs are considered to be the ideal source for clinical application and tissue engineering [4]. DPSCs’ cryopreserved character of the time-dependent manner is another advantage to its application [70]. As for the feasible availability, DPSCs could be obtained from orthodontic extraction teeth or wisdom teeth in a common surgical and non-invasive practice. Moreover, it can be easily passaged for more than 80 passages keeping the differentiation capacity [39, 40].

In order to better understand DPSCs’ character for further applications, many strategies have been developed to isolate DPSCs from adult dental pulp [68, 80]. One of the clinical studies has already adopted DPSCs for clinical alveolar bone reconstruction using patients’ own dental stem cells [3].

## Isolation, culture, and cryopreservation of DPSCs

In adult stem cell isolation, the key points are dissociation methods and selection markers. The dissociation method led the vitality of the stem cells, while the selection markers led the purity. Two main approaches have been applied for DPSCs dissociation, one is directly from pulp tissue (DPSC-ED) and the other one is outgrowth from tissue explants (DPSC-OG). Over 20 different enzymes and their combinations were considered during the DPSC dissociation methods. Collagenase I associated with dispase and collagenase alone were the most frequently used methods [16]. A recent research showed it will enrich more cells with CD146+, which were considered as the mainly DPSCs marker, as well as osteogenic and chondrogenic ability [14]. For the DPSC dissociation from the tissue explants outgrowth, although different enzymes showed different influences, studies claimed that the size of tissue fragments has no influence on osteoblast outgrowth [73]. By comparing DPSC-ED with DPSC-OG, it suggested that DPSC-ED have higher mineralization capacity while Hilkens and collaborators showed both DPSC-ED and DPSC-OG could successfully differentiate into adipogenic, chondrogenic, and osteogenic cell types [22]. However, it is related to the long migration time of cells from pulp tissue, so more than half studies adopted the enzymatic technique.

Unlike the dissociation method, the DPSC culture method still needs further development. The most common basal medium is α-MEM followed by DMEM. For the further application purpose, Serum-free media have been continuously tested for stem cell culture. Guo and his group established a chemically defined serum-free culture system for human dental pulp stem cells and found the serum-free Essential 8 medium might be applicable for hDPSCs culture in the future [81]. However, some researches indicated that these media do not adequately support DPSC proliferation and differentiation. As a consequence, various human blood derivatives have been proposed as alternatives to animal serum for stem cell culture, which includes autologous or allogenic human serum, human plasma, and human platelet lysates (PL) and their released factors. Marrazzo P and his group found that a low selected concentration of PL (1%) was able to support the growth and maintain the viability of the DPSCs in vitro [49]. Also, additional PL was shown as a suitable option for protocols promoting osteogenic and chondrogenic differentiation of DPSCs.

As mentioned before, DPSCs’ cryopreserved character is the necessary advantage for cell-based therapy. Gianpaolo Papaccio and his group demonstrated DPSCs and their osteoblast-derived cells can be long-term cryopreserved [61]. Lindemann and his group found that DPSCs were obtained from cryopreserved intact deciduous teeth without changes in the immunophenotypical characteristics and differentiation ability [47]. Nam Cong-NhatHuynh and his group revealed that controlled-rate freezing in 5% DMSO gave the highest rate of cell viability [37]. Recently, magnetic cryopreservation has been successfully used for tooth banking with satisfactory implantation outcomes [42].

## DPSCs differentiation

Differentiation ability is another key character of stem cell, so does DPSCs. As one kind of adult stem cells, the most key differentiation potential is the purpose tissue or cells itself. To DPSCs, it means odontoblasts. After transplanting into immune-compromised mice, human DPSCs will automatically differentiate into the dentin-like structure with odontoblast-like cells [20]. By seeding on chemically and mechanically treated dentin surface, DPSC-derived tissues also showed odontoblast-like morphology formation with dentinal tubule through scanning electron microscopy [24, 75]. Additionally, the increase of dentin matrix component-related genes, such as dentin matrix protein 1 (DMP-1) and dentin sialophosphoprotein (DSPP) expression double, confirmed odontoblasts differentiation results [11]. In the process of odontoblasts differentiation, research showed the notch signaling pathway [90] may help to induced angiogenesis and differentiate to regenerate vascularized dental pulp [41, 85].

DPSCs have also been proved to differentiate into other cell types including all three germ layers. The detailed information of differentiation methods and checking notes were shown in Table 1. Mesoderm lineage differentiation was well established including osteocytes, adipogenic, and chondrogenic. Experiments showed DPSC osteo-differentiation both in vivo and in vitro. Genetic profiles between DPSCs and normal osteoblasts identified functional gene activities changed including adhesion and cytoskeletal elements production regulation [6]. Adipogenic differentiation from hDPSCs has been confirmed by several studies, including direct culture in adipo-inductive medium supplied with dexamethasone [21, 33, 52]. By using hDPSCs from human unerupted third molars with completely formed crown but without well-developed roots, the differentiated cells were stained positively with Oil-Red-O and expressed adipocyte-specific genes such as PPAR-A2 and ap2 detected via RT-PCR analysis [82]. By ascorbate-2-phosphate and transforming growth factor (TGF)-b1 induction or co-cultured with human costal chondrocytes (CCs), the DPSCs will go chondrogenic differentiation and improve the cartilage formation.

**Table 1:** Detailed information about the differentiation of dental pulp stem cells

	Cell type	Time	Differentiation strategy	Detect methods	References
Entoderm	Liver cells	40 days	Factors inducing	In vitro	[17] [30]
Mesoderm	Melanocytes	120 days	Factors inducing	In vitro	[60]
	Chondrogenic cells	3 weeks	Factors inducing Co-cultured with human costal chondrocytes	In vitro	[58] [77] [9] [72] [76] [57] [43]
	Myogenic cells	1 month	Factors inducing	In vitro	[39]
	Adipocytes	3 weeks	Factors inducing	In vitro	[52] [58] [33] [21] [88] [56]
	Osteoblasts	3 months	Factors inducing	In vitro	[39] [17] [61]
	Osteocytes	3 weeks	Factors inducing	In vitro In vivo	[58]
Ectoderm	Odontogenic cells	4–8 weeks	Subcutaneous implantation	In vivo	[58] [20] [66] [24] [11] [74, 75]
	Schwann and neural cells	15 days	Factors inducing	In vitro In vivo	[20] [17] [58]

The ectoderm or endoderm lineage cells differentiated from DPSCs have also been reported. DPSCs express high expression of various neural crest-related and neural crest developmental genes since they are derived from neural crest origin [32, 52]. DPSC neurogenesis is highly related with FGF signal pathway. By inducing with bFGF, the neurogenic markers and neurosphere sizes of DPSCs have been upregulated. On the other hand, if inhibits FGF receptors, the neuronal differentiation of DPSCs will decrease.

A hepatic lineage of cells has been differentiated from human dental pulp cells although the purity was not very high [29]. More and more methods are tried in order to get purer hepatic lineage, and a novel protocol has been modified for hepatic differentiation in vitro from DPSCs and SHEDs. Moreover, their differentiation can last for a long time after 70 populations and DPSCs might not be as good as SHEDs considering as the hepatic progenitor source [30]. Besides, the CD117-positive cells may be used as the marker for hepatogenic lineage differentiation, which is adopted for future transplantations.

## Application of DPSCs and tissue engineering applications

### Application of DPSCs

DPSCs can be used in various aspects such as tissue engineering and regenerative medicine owing to their high proliferative and multilineage differentiated ability [25, 58]. It is an alternative choice for iPSC to solve the problems in re-programming and epigenetic changes [13, 79]. Dental stem cell therapy adopts the multidirectional differentiation character to reconstruct normal cell function or repair disease cells [7].

The first successful example is treating spinal cord injury (SCI) which leads to sensation loss and extremities paralysis. Comparing with BMSC and AMSC, DPSCs could enhance the survival rate of endogenous glia and neurons [65] owing to its secretion of NTF titres [50] after transplantation. DPSCs were also applied in treating traumatic brain injury (TBI) and stroke. In a focal cerebral ischemia rat model, DPSCs helped to improve forelimb sensorimotor function after transplantation. Rather than neurons, DPSCs could also contribute into glia, which may mediate paracrine pathway opposite to replacing the neurons that lost during ischemic damage directly [44]. Another evidence for improving TBI repair is that the pre-differentiated DPSC could migrate to different brain areas including the lesion region and then adopt a neuronal phenotype that expresses functional potassium and sodium currents [36]. Another popular application for stem cell regeneration is the treatment of retinal repair in ocular diseases. It has already been proved that DPSC can differentiate into photoreceptor phenotype when exposed to a conditioned medium of lesioned organotypic retinal cultures [5]. The animal experiment showed the possibility of human DPSC can decrease the RGF loss in glaucoma which elevated intraocular pressure [51]. It is even reported to treat radioactive esophageal injury by regenerating esophageal tissues [87].

Moreover, DPSCs may involve in deciduous teeth root reabsorption process [84]. Pierdomenico et al. think that DPSCs may have immunosuppressive activity but need future confirmation [62]. More and more studies begin to focus on DPSCs in recent years; thus, many breakthroughs were made in DPSC clinical application and researches while it is still in infancy. More theoretical mechanism and studies are needed for future applications, and lots of technical problems have not been solved. DPSCs cultured together with odontogenic cells via epithelial-mesenchymal interactions may help stem cells adapt to dental cell lineages and make the scaffold matrix become part of teeth [69].

Excitingly, DPSCs have been used in vivo and reported in many articles. Two systematic reviews [10, 53] were published to summarize and synthesize the information. One collected all the in vivo studies which used DPSCs to repair or regenerate non-dental tissues. From the data in 14 eligible studies including in 2309 papers, most of the DPSC application in vivo are successful, while it is still not guaranteed for clinical management [10]. The other one assessed in vivo research on DPSCs efficacy for bone regeneration in animal models. After assessing 17 individual studies, the authors draw conclusions that DPSCs were capable of regenerating the bone in vivo but still need more homogeneous studies to make a precise conclusion [53]. Moreover, Lei et al. carried out in vivo experiment and claimed that DPSCs maintain the MSC characteristics after in vivo implantation and more stable under in vivo conditions compared to PDLSCs [43]. Hilkens et al. evaluated the angiogenic potential of DPSCs in an in vivo model of dental pulp regeneration and demonstrated the successful formation of vascularized pulp-like tissue in 3D-printed scaffolds, which indicates a promising approach in dental tissue engineering [23]. Paino et al. conducted a research in vivo adopting human DPSCs fabricate vascularized woven bone tissue concluding that they can be used for customized regeneration [59]. Besides, a study discovered that 3 years after transplants in human mandibles, histological and in-line holotomography revealed that stem cells regenerated a compact rather than a spongy bone, which may have a positive clinical impact [18].

### Tissue engineering applications in stem cells

While the shortage of traditional cell culture limits the application of stem cell-based cell therapy, tissue engineering strategies were used to enhance DPSCs in vitro function. By mimicking the physicochemical and biological signal niche, combining the engineering and material methods [41, 54], and rebuilding the feature of destination tissue may be a natural way to help push the regeneration medicine field forward.

Usually, the basic tissue engineering method includes scaffold reconstruction, hydrogel matrix support, and artificial patterning design. These three methods always support each other to develop enhanced complex both in tissue structure and function. Limited by the weak mechanical properties of the hydrogel, scaffolds have usually been fabricated as the framework for cellular behavior and function. For regeneration medicine use, the first consideration of the scaffold material should be the character of non-toxic, less side effects, high biocompatibility, and low immunogenicity. For the engineering tissue preparation, the scaffold material needs to be extensive and the preparation process should be simple and repeatable, as well as environmentally friendly. Undoubtedly, all the above pose-specific problems and challenges for the development of tissue engineering scaffold materials indicate the direction.

Choosing biocompatible materials and designing mimic device will help to enhance cell interaction and stimulating spontaneously regeneration to format self-regulating tissue function, instead of artificially constructing complexity of living tissues ex vivo. The 3D geometrical features, mechanical property, surface feature, and other biocompatibility of materials influence cell adhesion, proliferation, differentiation, and pluripotency maintenance. The different cells in different surrounding materials are able to regulate self-gene expressions and secrete new ECM which will lead the other cells fate determination [45]. A well-designed device also has a similar function, for example, a novel, modular nerve-lengthening device with scaffold giving the imposition of moderate tensile for axonal outgrowth [8]. More and more studies seek to investigate the biological effects of the properties of biomaterials in TE, which is called material biology; it is a new concept draws from material science [45].

### Potential applications of DPSC combine with tissue engineering

Combined tissue engineering with DPSC, some approaches towards the regeneration medicine application have already been reported. Base on the serious of the disease and DPSCs’ characters, most of the applications focus on neurology, tooth or bone reconstruction, and angiogenesis, liver, esophageal, or bladder regeneration. Here, we list the examples for hDPSCs combined with tissue engineering in neuro-, bone, and dentin-pulp regeneration.

A study of 3D Floating Sphere Culture System provides a respectable microenvironment for hDPSCs to preserve their neuronal properties significantly compared to osteogenic and myogenic commitments [63]. If the neutrosphere strategy is the simplest application for tissue engineering, the reconstruction of the bone and dentin-pulp are the solid engineering work.

Previous studies have been well demonstrated the osteogenic differentiation capacity of DPSCs, including high expression of bone-specific markers [2]. Scaffold composition and surface properties play a critical role in the proliferation and differentiation of DPSCs. Collagen type I matrix could significantly improve mineral formation; moreover, hydroxyapatite (HA) and tricalcium phosphate (TCP) have been widely applied in increasing osteoconductive in the process of scaffold forming [46, 78]. After being seeded on 3D printing TCP/collagen hybrid for 3 weeks, DPSCs were able to pre-differentiated into osteoblast-like cells accompanying with activated ALP [15]. Also, DPSCs cultured on fibrin, hyaluronic acid, and PEA-C exhibited superior mineralization values than standard tissue culture on TCPs [1].

Root canal therapy is a common treatment for trauma and infection of adult pulp. After root canal therapy, the entire pulp was removed and often followed by tooth fracture and finally lead to loss of teeth. It is noteworthy that DPSCs have the capacity to generate dentin that rendered dentin-pulp regeneration possibility [20]. The process of generating dentin genesis includes odontoblastic deposition, vascularization, and neuron formation. It is reported that DPSCs could differentiate into functional odontoblasts and exhibit angiogenic potential that could be heightened by endothelial cells and endothelin-1 [12, 48]. In an artificial human root canal model, DPSCs in the empty root canal space can generate pulp-like tissue with well-established vascularity and that odontoblast-like cells produce dentin-like hard tissue on the dentinal walls [26].

Moreover, special growth factors and scaffold materials are important factors for improving functional effectiveness in dentin-pulp TE. According to the report, DPSCs that are transplanted with stromal cell-derived factor 1 (SDF1) in a collagen scaffold could complete pulp regeneration in a canine pulpitis model [27]. In addition, regenerated pulp tissue induced by granulocyte colony-stimulating factor (G-CSF) treatment was formed in the coronal part and prevented microleakage up to day 180 in a dog pulp-ectomized tooth model [28]. Reciprocally, a recent research put scaffold-free 3D DPSC with sheet-like aggregate shapes with a thermo-responsive hydrogel into the human tooth root canal and implanted subcutaneously into immunodeficient mice. After 6-week implantation, pulp-like tissues with rich blood vessels were observed and blood vessel-rich pulp-like tissues can be formed with DPSCs without adding growth factors and scaffolds [31].

## Conclusion and challenges

As a promising cell source for numerous and varied regenerative medicine applications, DPSCs become one of the target adult stem cells which need to further understand and develop. Although some achievements have been made in the study of DPSC, several challenges remain to be solved. For example, as the main problem in all kinds of stem cells transplantation, low survival rates, especially low long-time survival rates, were still a key concern for whether the recover function really comes from DPSCs’ tissue function rebuild or secretion effect [44, 55]. Multifield cooperation is urgently needed to dig into the mechanism as well as the technic related to DPSC differentiation and artificial tissue construction. More importantly, as most of the studies conducted on animal models, more clinic-related experiments are necessary to evaluate the efficacy of the procedures in regenerating defects in human.

## Abbreviation

BMSCs: Bone marrow stem cells
CCs: Costal chondrocytes
DMP-1: Dentin matrix protein 1
DMSO: Dimethyl sulfoxide
DPSCs: Dental pulp stem cells
DSPP: Dentin sialophosphoprotein
FGF: Fibroblast growth factor
G-CSF: Granulocyte colony-stimulating factor
hDPSCs: Human dental pulp stem cells
IDPSCs: Immature dental pulp stem cells
PL: Platelet lysates
SC: Stem cell
SCI: Spinal cord injury
SDF1: Stromal cell-derived factor 1
SHEDs: Stem cells from human exfoliated deciduous
